The article "Impact of Aging in Microglia-Mediated D-Serine Balance in the CNS" was published in 2018. Journal: Mediators Inflamm.

# Impact of Aging in Microglia-Mediated D-Serine Balance in the CNS

**DOI:** 10.1155/2018/7219732

**Published:** 2018-09-27

**Authors:** Sebastián Beltrán-Castillo, Jaime Eugenín, Rommy von Bernhardi

**Affiliations:** ^1^Departamento de Neurología, Escuela de Medicina, Pontificia Universidad Católica de Chile, Santiago, Chile; ^2^Departamento de Biología, Facultad de Química y Biología, Universidad de Santiago de Chile, Santiago, Chile

## Abstract

A mild chronic inflammatory state, like that observed in aged individuals, affects microglial function, inducing a dysfunctional phenotype that potentiates neuroinflammation and cytotoxicity instead of neuroprotection in response to additional challenges. Given that inflammatory activation of microglia promotes increased release of D-serine, we postulate that age-dependent inflammatory brain environment leads to microglia-mediated changes on the D-serine-regulated glutamatergic transmission. Furthermore, D-serine dysregulation, in addition to affecting synaptogenesis and synaptic plasticity, appears also to potentiate NMDAR-dependent excitotoxicity, promoting neurodegeneration and cognitive impairment. D-serine dysregulation promoted by microglia could have a role in age-related cognitive impairment and in the induction and progression of neurodegenerative processes like Alzheimer's disease.

## 1. Introduction

Microglia are the main innate immune effector cells of the brain and the main generator of inflammatory cytokines and reactive oxygen species in the central nervous system (CNS) [1–3]. It is debated whether microglia have a beneficial or a deleterious role under pathological conditions. In pathological conditions, a large spectrum of beneficial microglial phenotypes releasing anti-inflammatory cytokines and neurotrophic factors that contribute to tissue repair and neuroprotection against injury or infections can be found. However, they coexist with noxious microglial phenotypes that release reactive oxygen species, proteinases, and inflammatory cytokines contributing to neuronal damage [4]. Moreover, microglial activation under physiological conditions, in addition to promote the removal of noxious stimuli and the activation of reparative mechanisms, has also the potential of modifying D-serine levels.

D-serine is a dextro amino acid, which is a coagonist of the glycine strychnine-insensitive site of the glutamate N-methyl-D-aspartate receptor (NMDAR) [5, 6], found in neurons, astrocytes, and microglia [7–11]. Increased levels of D-serine can potentiate glutamate transmission, increasing synaptic activity on one hand, but it potentially can also facilitate glutamate-induced excitotoxicity on the other.

The article "Impact of Aging in Microglia-Mediated D-Serine Balance in the CNS" was published in 2018. Journal: Mediators Inflamm.

Aging is associated with morpho-functional changes in neurons and glial cells. Changes in the activation and regulation of microglia can promote a chronic inflammatory state [12] in the CNS. Aged microglia show cellular, molecular, and functional differences compared with microglia from young individuals, including morphological changes suggesting they are activated even under nonstimulated conditions [13], elevated basal levels of proinflammatory cytokines such as interleukin 6 (IL6) and IL1*β* [14, 15], and increased reactive oxygen species (ROS) production [16]. They have also a decreased ability to upregulate the phagocytosis of *β*-amyloid (A*β*) in response to inflammatory stimulus [17–19] and an impaired regulation of their inflammatory activation that depends on changes of transforming growth factor *β*1 (TGF*β*1) signaling [16].

Here, we describe evidence that aged microglia can promote D-serine dysregulation in the CNS and discuss how the imbalance between D-serine and other regulatory mechanisms can result in glutamate and D-serine-mediated impairment of synaptic plasticity and neurodegeneration, which can result in cognitive impairment. Those mechanisms could be involved in neurodegenerative diseases in which aging is the main risk factor, such as late onset Alzheimer's disease (LOAD) [12].

## 2. D-Serine in the CNS

D-serine has emerged as a novel regulatory factor giving a new twist to glutamatergic transmission and how aging can affect it. D-serine is an effective agonist of the strychnine-insensitive glycine site of the glutamate NMDAR [5, 20] detectable at substantial quantities in the rat brain tissue [21], exhibiting a brain distribution similar to that of NMDAR [22], and showing age-dependent changes in its anatomical distribution closely correlated with that of NMDAR [23].

In the CNS, D-serine is found in astrocytes, radial glial cells, neurons, and in quiescent and activated microglia [7–11]. D-serine is synthetized by isomerization of L-serine, in a reaction catalyzed by the enzyme serine racemase [24, 25], which, in addition to synthesize D-serine, also catalyzes the *α*,*β*-elimination of water from L-serine or D-serine to produce pyruvate and ammonia [26] (Figure 1). D-serine is preferentially degraded through oxidation by the enzyme D-amino acid oxidase [27] and also by the serine racemase-mediated water *α*,*β*-elimination induced by elevated intracellular D-serine levels [26] (Figure 1). Serine racemase is expressed by many CNS cells, including pyramidal neurons in the cerebral cortex, gamma-aminobutyric acid (GABA) ergic medium-spiny neurons in the striatum, cerebellar GABAergic Purkinje cells [28], vestibular nuclei neurons [29], astrocytes from the caudal medulla oblongata [11], telencephalon, and the CA1 region of the hippocampus [22], and neurons and astrocytes from the retina [30, 31]. However, which cells are the principal source of D-serine release in the CNS is still controversial [32, 33]. The predominant source appears to depend on the CNS area, function, developmental stage, and inflammatory state [7, 8, 11, 31, 34, 35].

The article "Impact of Aging in Microglia-Mediated D-Serine Balance in the CNS" was published in 2018. Journal: Mediators Inflamm.

The “serine neuron-astrocytes shuttle” hypothesis explains the relation of D-serine synthesis in neurons and astrocytes. Here, on the one hand, neuronal D-serine production requires the production of L-serine by astrocytes because the enzyme 3-phosphoglycerate dehydrogenase that catalyzes the synthesis of L-serine from glucose is localized almost exclusively in astrocytes [36–38]. On the other hand, neuronal D-serine is released from neurons by depolarization and it is uptake and stored by astrocytes, until D-serine is required for modulating the glutamatergic NMDA transmission [39]. However, this hypothesis does not consider alternative sources of D-serine like microglia, in which both serine racemase and D-serine are also found. In fact, activation of microglia by lipopolysaccharide (LPS), the amyloid precursor protein (APP), and amyloid *β*-peptide (A*β*) induces the upregulation of serine racemase and increases the release of D-serine [7, 35]. The mechanism of D-serine release by microglia is still unclear, whereas D-serine release by astrocytes has been explored and includes Ca^2+^- and SNARE-dependent exocytosis, as well as other nonexocytic mechanisms, such as volume-regulated anion channels (VRAC), alanine–serine–cysteine transporter (ASCT), and gap junction hemichannels [11, 40–48].

D-serine participates in multiple processes, including synaptic plasticity [5, 49], cell migration, synaptogenesis [22, 50], and in homeostatic functions, as a mediator of hypercapnia-induced respiratory response [11]. D-serine production and release appear to be closely regulated, and its concentration kept in a narrow range. Dysregulation of D-serine may lead to pathology. Abnormally increased levels of D-serine are associated with NMDAR-mediated neurotoxicity [9, 51, 52], whereas abnormally decreased levels are associated with impairments in functional plasticity and memory deficits [53]; as we will discuss later.

## 3. Function of Microglia in the CNS

Microglia are highly plastic cells and can respond to a broad spectrum of stimuli, which includes infection, ischemia, inflammation, cell death, trauma, and toxins [54]. Activated microglia change their morphology and their functional properties, generating ROS, nitric oxide (NO∙) [55], and several inflammatory and regulatory cytokines, including interleukin 10 (IL10), IL1*β*, IL6, tumor necrosis factor *α* (TNF*α*), and interferon *γ* (IFN*γ*) [12, 15, 16, 56–60] in addition to D-serine [7, 34]. Microglia activation promotes changes in the environment, affecting the function of neighbor cells. On bases of functional properties, a wide activation spectrum has been characterized for microglia, similar to that described for macrophages [61]. Two phenotypic extremes are recognized: the M1-like profile, corresponding to cells that are very proinflammatory and have poor phagocytic activity, and the M2-like profile, evidenced by cells that are anti-inflammatory, neuroprotective, and show a robust phagocytic activity [61]. The M2-like profile microglia are most frequently induced under homeostatic conditions through immunomodulation by astrocytes and neurons [62]. In contrast, a shift from a M2-like to a M1-like profile is often observed in several neurodegenerative diseases, including Alzheimer's disease (AD) [63].

The article "Impact of Aging in Microglia-Mediated D-Serine Balance in the CNS" was published in 2018. Journal: Mediators Inflamm.

TGF*β*1 signaling mediates, at least in part, the immunomodulation of microglia by neurons and astrocytes [19, 64, 65]. TGF*β*1 plays a relevant neuroprotective role, attenuating and restricting the duration of neuroinflammation and neurotoxicity [64, 65]. The neuroprotective effect of TGF*β*1 is mainly mediated by the activation of the Smad pathway (TGF*β* canonical signaling) in microglia, which decreases the release of proinflammatory cytokines, ROS, and NO∙ [60, 64] and promotes phagocytosis and A*β* clearance by microglia [66]. However, TGF*β*1 activates also non-Smad-dependent signaling pathways, including MAPKs (ERK, P38, and JNK) and PI3K [60, 67, 68]. With exception of the ERK pathway, which under certain conditions activates neuroprotective effects [69], the activation of signaling mediated by the other MAPKs and PI3K potentiates neuroinflammatory activation [12]. Therefore, microglia play an important role of protection against infection and repair of the damage produced by injury of the CNS. However, they must accomplish their action under the modulation exerted by neurons and astrocytes through an adequate functional signaling.

### 3.1. Participation of Microglia on D-Serine Regulation

D-serine levels are not homogeneous among different CNS areas. The level of D-serine is in the order of 200–300 pmoles per milligram of tissue in the hippocampus, frontal cortex, and cerebellum, 20-fold higher than in the pancreas, lung, or testis and almost 100-fold higher than in muscle [70]. In the hippocampus, D-serine and serine racemase are predominantly observed in the neuron-rich pyramidal cell- and in the granule cell-layers [71]. A neuronal tonical release of D-serine [71] that maintains a concentration of free D-serine at around 0.3 *μ*M [70] allows synaptic potentiation and plasticity. However, in mice models of hippocampal synaptic damage secondary to trauma (controlled cortical impact: CCI), a switch between neuron and astrocyte production is observed: serine racemase is downregulated in neurons and upregulated in astrocytes [71]. Thus, the content of D-serine is reduced in neurons, but it is increased in astrocytes. The CCI-induced enhancement of D-serine release from astrocytes is detrimental for synaptic potentiation and plasticity [71].

The article "Impact of Aging in Microglia-Mediated D-Serine Balance in the CNS" was published in 2018. Journal: Mediators Inflamm.

We propose that microglia are also contributing to the increase of free D-serine as consequence of their activation by inflammatory stimuli. Thus, in addition to releasing pro- and anti-inflammatory cytokines and chemokines [72], microglia activation also induces the release of excitatory amino acids, including glutamate and D-serine [34, 35, 73]. The levels of serine racemase are increased in response to A*β* peptide, lipopolysaccharide (LPS), or secreted amyloid precursor protein (sAPP), associated with an increased expression of serine racemase [34, 35]. The amount of D-serine released by these stimuli can be neurotoxic for hippocampal neurons in culture [7].

### 3.2. Microglia Impairment in Aging

Aging is a normal dynamic process in life, characterized by the development of a mild inflammatory environment in the organism and a progressive deterioration of some physiological functions, largely attributable to the loss or dysfunction of cells, even in the absence of overt disease [74]. This deterioration and loss of function also affects the CNS, where it is particularly dramatic [75, 76] and can include impairments in behavior, cognitive ability, learning, and memory [77]. Aging is also associated with changes in the immune system in a phenomenon known as immunosenescence [78]. Immunosenescence is induced by cumulative low-level inflammation, which induces changes in gene expression related to immune response and inflammation [79, 80], resulting in an exacerbated inflammatory response against stressors, which could facilitate the onset and progression of neurodegenerative diseases [81–83]. The aged or “senescent” microglia show exacerbated reaction to minor injuries or mild stimuli, with a potentially damaging response [60], generating cytotoxicity and promoting neurodegenerative changes [12]. Unlike young microglia, aged microglia show increased production of ROS and inflammatory cytokines, with decreased NO^·^ production [19], decreased ability to phagocytose A*β* [17], and reduced LPS- or TGF*β*-induced A*β* phagocytosis by microglia [19]. Those facts led us to reconsider the real role of A*β* in AD pathology, changing our focus from the “amyloid cascade hypothesis” in which A*β* accumulation is the pathogenic cause of AD, and neuroinflammation is its consequence [84–86], to the “glial dysfunction hypothesis” [60, 82]. In the “glial dysregulation hypothesis”, the genesis of AD is placed at the dysfunction of the innate immune response associated with chronic neuroinflammation and aging [82, 87, 88].

The article "Impact of Aging in Microglia-Mediated D-Serine Balance in the CNS" was published in 2018. Journal: Mediators Inflamm.

Dysfunction of microglia can result, at least partly, in deregulation of TGF*β*1 signaling, one of the main regulatory cytokines in the brain [89]. The neuroprotective regulation of microglia activity by TGF*β*1 is mediated mainly by the activation of Smad3 and, to a lesser extent, by activation of ERK [69, 90]. In addition, TGF*β*1-activated PI3K and MAPK signaling could potentiate neuroinflammation [12]. A reduced activation of TGF*β*1-Smad3 signaling in microglia has been reported in 12-month-old adult mice compared with juvenile mice [19, 60], regardless of the fact that TGF*β*1 levels are elevated at that age. In fact, elevated levels of TGF*β*1 has been reported in AD patients [91, 92]. The reduced response of microglia to TGF*β*-Smad3 modulation could contribute to maintain a chronically activated microglia, increasing cytotoxicity and impaired uptake of A*β* [82, 93]. Thus, impairment of the innate immune response associated with aging-related changes in regulatory signaling could be the cause, and not a consequence, for the onset of neurodegenerative processes.

## 4. Role of D-Serine in CNS Development and CNS Levels in Aging

D-serine level in the CNS changes during development and aging. At early development stages, a transient increase on NMDAR activity [94] matches with a transient rush of D-serine production. Healthy newborn children have an elevated cerebrospinal fluid (CSF) D-serine level that is rapidly reduced during the first year of life and reaches 15% of the initial concentration at 3 years of age [95]. The elevated level of D-serine at early age has been associated with brain development, and its deficit is associated with alterations of normal brain development program. For example, 3-phosphoglycerate dehydrogenase deficient children show a severe but treatable disorder of serine synthesis, characterized by microcephaly, psychomotor retardation, and seizures [96]. Prenatal treatment with D-serine allows a nearly normal CSF D-serine level and an adequate clinical phenotype at birth [95].

D-serine has been also described in the development of the rat vestibular nuclei because it is a model of the vestibular plasticity mediated by glutamatergic AMPA and NMDAR neurotransmission observed in the posttrauma vestibular compensation [97]. Here, high expression of serine racemase and increased levels of D-serine are detected mainly in glial cells from birth until P21, with a peak at P7. After P21, both D-serine and serine racemase are reduced in glial cells at the vestibular nuclei, and high content of D-serine switches from glial cells to neuronal cell bodies and dendrites mostly because of an increased expression of glial D-amino acid oxidase at mature stages [29]. The early postnatal period with high D-serine level in glia coincides with a period of intense plasticity, synaptogenesis, and maturation at the vestibular nuclei, suggesting the existence of distinct functional roles for D-serine throughout development.

The article "Impact of Aging in Microglia-Mediated D-Serine Balance in the CNS" was published in 2018. Journal: Mediators Inflamm.

In other brain areas, D-serine level decreases in aging, and its reduction is associated with age-related memory impairment [98]. In the hippocampus of 24–29-month-old rats, both D-serine and serine racemase levels are decreased [8, 99]. In contrast, in a model of healthy aging like the Lou/C/Jall rat strain that preserves its cognitive function, D-serine and serine racemase levels are not affected by aging [100]. The preservation on memory and the resistance to age-related long-term potentiation (LTP) deficit [101, 102] observed in old Lou/C/Jall rats have been associated to their preference for low-calories food [103]. The caloric restriction reduces the generation of reactive oxygen species [104, 105], which in turn contributes to avoid the induction of a proinflammatory environment that favors the functional impairment of microglia [12]. As part of their functional impairment, the microglia-related dysregulation of D-serine [7, 34, 35] contributes to neurodegeneration and cognitive impairment [106].

The decrease of D-serine during aging has been also associated with an increase on mitochondrial carboxylate pyruvate enzyme expression impairing the modulation of NMDAR by D-serine secreted by astrocytes [98] and to the reduction of serine racemase expression in the hippocampus [99]. As mentioned for the vestibular nuclei, the levels of D-amino acid oxidase, the enzyme that degrades D-serine, can change in various brain areas during aging [107] and, therefore, affect D-serine level. In dementia patients, the severity of the cognitive deficit can be correlated with increased D-amino oxidase blood level [108].

How much of the changes in D-serine level during aging are determined by microglial cell actions has not been elucidated. However, we speculate that age-dependent changes on microglia regulation results in neuroinflammation and increased oxidative stress, which in turn activate production of D-serine by astrocytes and neurons [33, 71, 109–112]. Thus, aging on the one hand can promote overactivation of glutamatergic by increased D-serine level and on the other result in impaired activation. We will further discuss these mechanisms in the next section.

The article "Impact of Aging in Microglia-Mediated D-Serine Balance in the CNS" was published in 2018. Journal: Mediators Inflamm.

### 4.1. How Age-Related Impairment of Microglia Can Result in D-Serine Dysregulation

Both abnormally increased and decreased levels of D-serine are potentially deleterious for brain function. Although a reduction of D-serine levels has been preferentially reported [98] and associated with cognitive impairment in normal aging, we propose that persistent inflammatory activation of microglia in pathological aging leads to abnormally increased levels of free D-serine that may generate glutamate-mediated neurotoxicity [9, 51, 52] and impairment of the glutamate and D-serine-mediated plasticity. The resulting neurocognitive deficit contributes to the emergence of neurodegenerative changes. During aging, inflammation promotes changes in microglial regulation, increasing their reactivity and favoring a cytotoxic in contrast to a neuroprotective environment [12]. As mentioned in previous sections, modifications on the D-serine-mediated glutamatergic transmission associated with aging include changes in the expression of serine racemase and D-amino acid oxidase as well as in D-serine content. Serine racemase and D-serine are detectable in quiescent and increase when microglia are activated [34, 35]; the proinflammatory brain environment observed in aged individuals will stress overactivated or dysfunctional microglia, further promoting the production and release of gliotransmitters and neurotransmitters, including D-serine, by astrocytes and neurons [110–112].

The age-dependent changes in microglial TGF*β* signaling could also contribute to D-serine dysregulation because of molecular elements shared by TGF*β* signaling and serine racemase regulation [34, 113–115]. One is the Protein Interacting with C Kinase-1 (PICK1), a scaffold protein that plays a role in controlling the traffic of multiple membrane receptors and acts as a regulator of phagocytosis and oxidative stress in microglia [116, 117]. Elevated levels of TGF*β* promote the activation of PICK1, promoting the internalization, ubiquitination, and degradation of the TGF*β*1 receptor (TGF*β*R1) through a caveolin-dependent pathway, reducing the activation of the Smad-dependent pathway [113]. PICK1 also interacts with serine racemase [114], being a tag for PKC*α* activity in the reduction of serine racemase activity by phosphorylation in astrocytes and neurons [115]. Interestingly, imbalance among several PICK1 partners has been associated with induction of neurodegenerative diseases [118]. Another common element is Jun N-terminal kinase (JNK), which is involved in noncanonical TGF*β* signaling. In inflammation induced by LPS, activation of JNK phosphorylates c-JUN, activating the activator protein 1 (AP-1) and inducing the expression of the serine racemase gene [34]. The fact that the activation of JNK is part of TGF*β* activation raises the possibility that serine racemase expression can be regulated at least partly by TGF*β*. In addition, TGF*β* and D-serine also have a functional relationship in synaptogenesis.

The article "Impact of Aging in Microglia-Mediated D-Serine Balance in the CNS" was published in 2018. Journal: Mediators Inflamm.

### 4.2. D-Serine in Synaptogenesis

During embryonic development, astrocytes release TGF*β* that activates TGF*β*R1, inducing the release of D-serine by astrocytes and neurons. The released D-serine participates in the induction of synaptogenesis in cortical neurons in culture [50]. The synaptogenic effect induced by TGF*β* in cortical neurons is abolished by D-amino acid oxidase reduction of endogenous D-serine or serine racemase knockdown with specific short hairpin RNAs (shRNAs), suggesting a direct relationship between D-serine-mediated and TGF*β*-induced synaptogenesis [50].

In CNS development, D-serine shapes synaptogenesis and neuronal circuitry through activation of NMDAR. D-serine is a key player in astrocyte-mediated LTP associated with hippocampal plasticity [119]. This role is particularly important at early stages, where an elevated concentration of D-serine [95, 120] encounters a transient elevated activity of NMDAR [94]. In murine P19 cells, an embryonic carcinoma cell line that can be differentiated to resemble neurons with functional glutamatergic receptors [121], D-serine induces synaptogenesis and serine racemase is very active [122]. D-serine released by astrocytes acts also as a chemokine for migration of granule cells in the cerebellum [123], and, at embryonic and early postnatal development, its decrease compromised the adequate lamination of the cerebellar cortex [124].

The loss of astrocyte function induced by sodium fluoroacetate, a selective metabolic inhibitor of astrocytes, reduces LTP in the hippocampus and impairs learning and memory in adult rats but can be rescued by D-serine supplementation [125]. Finally, as mentioned above, the decrease of D-serine levels in aging, in special that released by astrocytes, is associated with age-related memory impairment [98]. These results, together with those showing the maintenance of serine racemase and D-serine levels in healthy aging models [126], suggest a pivotal role of D-serine in the induction and conservation of synapses. The role of D-serine in synaptogenesis is likely to remain active, although less robust than in prenatal development, into adulthood and beyond because the shaping of neural networks continues throughout life.

The article "Impact of Aging in Microglia-Mediated D-Serine Balance in the CNS" was published in 2018. Journal: Mediators Inflamm.

Microglia participate actively in synaptic regulation through various mechanisms. They participate in the formation of filopodia in somatosensory cortex by direct contact with dendrites [127], in synaptic pruning in the retinogeniculate system through CR3/C3-dependent phagocytic signaling [128], and in the formation of learning-dependent synapses in mice through brain-derived neurotrophic factor (BDNF) [129]. In addition, a microglial-dependent mechanism for synaptogenesis or synapsis pruning involving glutamate-D-serine-NMDAR signaling cannot be ruled out.

### 4.3. D-Serine as Inductor of Neurodegeneration

D-serine may promote NMDAR-dependent excitotoxicity, and overactivation of NMDAR can induce cell death [130], playing a role in neurodegeneration. However, NMDAR is also pivotal in neural plasticity. The localization hypothesis of NMDAR function proposes that functional outcomes are determined by NMDAR localization: whereas NMDARs localized outside synapses play a role in neurotoxicity; those localized in synapses would promote plasticity [131, 132]. Although extra synaptic and synaptic NMDARs are gated by different endogenous coagonists, glycine acting at extra synaptic NMDARs and D-serine at synaptic NMDARs [133], D-serine appears to be the dominant coagonist in NMDAR-mediated neurotoxicity in the hippocampus. This specific distribution opens the possibility to develop therapies to reduce the excessive activation of extra synaptic NMDAR. However, this segregation is not absolute. Both the long-term depression (which also contributes to plasticity) and the NMDAR-dependent excitotoxicity depend on the magnitude and duration of synaptic and extra synaptic activation of NMDAR [133, 134]. On the other hand, a probable contribution of D-serine from other sources, such as the microglia in the brain, has not been considered into the hypothesis.

During ischemia, microglia are activated and the extracellular concentration of D-serine increases in the cerebral cortex [135], promoting neuronal death mediated by NMDAR overactivation. Neuronal death can be avoided by reducing the endogenous D-serine by inducing D-amino acid oxidase [52, 136]. Similarly, D-serine synthesis and release by astrocytes and microglia [7, 34, 35] are increased at early inflammation stages in the spinal cord [137]. In addition, systemic inflammation generated by streptozotocin treatment contributes to diabetic retinopathy in Sprague-Dawley rats, inducing type I diabetes mellitus, neurodegeneration of the retinal ganglion cell layer associated with excitotoxity mediated by NMDAR overactivation [138], elevated expression of serine racemase in the retina, and a significant elevation of glutamate and D-serine levels in aqueous humor [139]. Interestingly, the neurodegeneration of the retina could be attenuated by the suppression of serine racemase activity [140]. Therefore, we can speculate that under inflammatory conditions, such as those induced by trauma, infection, or ischemia, microglia or other cells activated by them could increase the levels of free D-serine, promoting an uncontrolled activation of synaptic and extra synaptic NMDAR and inducing neuronal damage. Similarly, in aged individuals, the basal inflammatory conditions could facilitate the abnormal NMDAR activation.

The article "Impact of Aging in Microglia-Mediated D-Serine Balance in the CNS" was published in 2018. Journal: Mediators Inflamm.

### 4.4. D-Serine Level in AD

A postmortem study comparing D-serine level in the brain parenchyma from AD patients with nondemented individuals showed that AD patients had 2-, 3-, and 5-fold more D-serine in the hippocampus, cerebral cortex, and CSF, respectively [141]. Those results support the notion that neurobehavioral deficit at early stages of AD could depend on the impairment in synaptogenesis and functional plasticity mediated by D-serine, and later in the progression of the disease, on NMDAR-activated neurotoxicity. However, other studies report only mild increases in D-serine level in the CSF and frontal cortex from patients with AD or with Lewy bodies dementia [142, 143] or even a slight decrease in D-serine level in the serum of patients with this pathology [144]. These controversial results may depend on differences in the stage of progression of the disease.

Diagnosis of AD is done when damage is advanced. Nevertheless, the cognitive impairment observed in AD patients could depend, at least partly and in early stages, on impairments in synaptogenesis and functional plasticity and only later in damage depending on NMDAR-mediated neurotoxicity and promotion of neuronal death mediated by D-serine.

## 5. Concluding Remarks

In this work, we have discussed the physiological roles of D-serine in the brain and how it may contribute in the induction of neurodegenerative changes. We discussed how chronic inflammation may promote changes in microglial activation and regulation, promoting their increased reactivity, and a cytotoxic instead of a neuroprotective activation. Aged microglia, more inflammatory and less sensitive to TGF*β* regulation, can contribute to elevate D-serine levels in the brain (Figure 2), as they enhance serine racemase expression and D-serine release during inflammatory activation. The abnormal increase on free D-serine by overactivated microglia can potentiate glutamate-mediated neurotoxicity and impair glutamate-mediated plasticity. Thus, we hypothesize that the functional impairment of aged microglia results in D-serine dysregulation contributing to induction of neurodegenerative diseases like AD.

The article "Impact of Aging in Microglia-Mediated D-Serine Balance in the CNS" was published in 2018. Journal: Mediators Inflamm.

## Figures and Tables

**Figure 1:** D-serine synthesis and degradation. D-serine is synthetized by isomerization of L-serine in a reaction catalyzed by the enzyme serine racemase which, in addition, also catalyzes the *α*,*β*-elimination of water from L-serine or D-serine to produce pyruvate and ammonia. Although serine racemase also has the potential to degrade D-serine through *α*,*β*-elimination of water, it is preferentially degraded through oxidation by the enzyme D-amino acid oxidase, generating hydroxypyruvate, peroxide, and ammonia.

**Figure 2:** Impact of aging in microglial function and release of D-serine. In aging, a mild chronic inflammation promotes dysfunction of microglia and their cytotoxic activation. In contrast to young microglia, aged microglia show changes in TGF*β*1-Smad signaling that promote an inflammatory microglial phenotype. They release decreased levels of anti-inflammatory cytokines and high levels of proinflammatory cytokines and D-serine. The inflammatory environment together with increased levels of free D-serine could induce impairment in synaptogenesis and synaptic plasticity and contribute to neurodegeneration.
